This article has been retracted.

# Short-Term and Long-Term Curative Effect of Partial Hepatectomy on Ruptured Hemorrhage of Primary Liver Cancer after TAE

**DOI:** 10.1155/2022/2484418

**Published:** 2022-07-05

**Authors:** Xiulin Xiao, Lin Zhou, Long Zhang, Zhiyuan Xu, Qixin Dai, Xiaohong Deng

**Affiliations:** Department of Hepatopancreatobiliary Surgery, Ganzhou People's Hospital, Ganzhou, Jiangxi 341000, China

## Abstract

**Objective:**

To observe the short-term and long-term curative effects of partial hepatectomy on ruptured hemorrhage of primary liver cancer after transcatheter arterial embolization (TAE).

**Methods:**

A total of 150 patients with primary liver cancer treated in the hospital were enrolled as research objects between February 2018 and February 2021, including 75 cases undergoing TAE in the TAE group and the other 75 cases undergoing elective partial hepatectomy after TAE in the combination group. The surgical related indexes (leaving bed time, discharge time, success rate of hemostasis, lesion clearance rate), mean arterial pressure (MAP), heart rate (HR), hemoglobin, and liver function indexes (serum alpha-fetoprotein (AFP), albumin (ALB), total bilirubin (TBIL)) before and after treatment, postoperative complications, survival rate, and recurrence rate at 1 year after surgery between the two groups were compared.

**Results:**

Compared with the TAE group, hospitalization time was shorter (*P* < 0.05), the success rate of hemostasis and lesions clearance rate were higher in the combination group (*P* < 0.05). After surgery, levels of HR and serum AFP were significantly decreased, while levels of MAP, hemoglobin, serum ALB, and TBIL were significantly increased in both groups. The levels of HR and serum AFP in the combination group were lower than those in the TAE group, while levels of MAP, hemoglobin, serum ALB, and TBIL were higher than those in the TAE group (*P* < 0.05). There was no significant difference in the incidence of postoperative complications between the two groups (*P* < 0.05). Compared with the TAE group, the recurrence rate was lower, and the survival rate was higher in the combination group at 1 year after surgery (*P* < 0.05).

**Conclusion:**

Partial hepatectomy can effectively improve hemostatic effect and liver function in ruptured hemorrhage of primary liver cancer after TAE, increase survival rate, and reduce postoperative recurrence rate.

## 1. Introduction

Primary liver cancer is a malignant tumor that occurs in hepatocytes or intrahepatic bile duct epithelial cells and is prone to intrahepatic hematogenous metastasis [1]. Rupture and hemorrhage of liver cancer is a serious complication of primary liver cancer, with a mortality rate as high as 25% to 75%, which is the fourth leading cause of death in patients with liver cancer [2]. Due to the rapid onset of the disease, and because it is often accompanied by shock, its treatment is difficult, and the prognosis is poor. If it is not actively treated, it may accelerate the death of patients. In recent years, with the development and popularization of interventional techniques, interventional hemostasis has been widely used in the treatment of ruptured hemorrhage from liver cancer. Transcatheter arterial embolization (TAE) is an interventional minimally invasive surgical method, which is widely used in the treatment of ruptured hemorrhage of liver cancer. A study [3] reported that for patients with ruptured and hemorrhagic hepatocellular carcinoma who could not be resected by emergency surgery, the application of TAE for hemostasis was effective and could prolong the postoperative survival time of the patients. At present, there are many reports about liver resection and TAE in the treatment of primary liver cancer spontaneous rupture and hemorrhage [4–6], but there is no unified guideline for the selection of surgical methods for ruptured hemorrhage of primary liver cancer. Therefore, this study explored the short-term and long-term curative effects of partial hepatectomy on ruptured hemorrhage of primary liver cancer after TAE in order to provide more evidence-based data support for the selection of surgical options for the clinical treatment of ruptured hemorrhage of primary liver cancer. The study was reported as follows.

## 2. Materials and Methods

### 2.1. General Information

A total of 150 patients with primary liver cancer diagnosed and treated in our hospital from February 2018 to February 2021 were selected as the research objects, including 75 cases undergoing TAE in the TAE group and the other 75 cases undergoing elective partial hepatectomy after TAE in the combination group. Inclusion criteria were meeting the criteria of the primary liver cancer [7], abdominal contrast-enhanced CT showing liver cancer ruptures and hemorrhages with abdominal and pelvic cavity and blood, and the diagnostic paracentesis not coagulating; meeting TAE or partial indications for hepatectomy; liver function grade *A* or *B*; and clinical data including postoperative follow-up data were kept intact. Exclusion criteria were severe heart, brain, liver, kidney dysfunction, coagulation dysfunction; previous history of abdominal surgery; distant metastasis or multiple intrahepatic metastasis of liver cancer; and advanced liver cancer. TAE group (75 cases): 43 males and 32 females; aged 43–71 years, mean (56.27 ± 6.03) years old; 71 cases were hepatitis B positive; 66 cases were alpha-fetoprotein (AFP) positive; Child-Pugh grade included grade A (62 cases), grade B (13 cases); the tumor diameter was 6.45–12.53 cm, with an average of (9.24 ± 1.36) cm; tumor sites: left lateral lobe, left medial lobe, right anterior lobe, and right posterior lobe were 19, 22, 25, and 9 cases, respectively; and 31 cases of admission combined with shock. Combination group (75 cases): 40 males and 35 females; aged 43–76 years, mean (56.92 ± 5.99) years old; 71 cases of hepatitis *B* positive; 67 cases were alpha-fetoprotein (AFP) positive; Child-Pugh grade included grade *A* (65 cases), grade *B* (10 cases); the tumor diameter was 6.38–11.60 cm, with an average of (8.87 ± 1.34) cm; tumor sites: left lateral lobe, left medial lobe, right anterior lobe, and right posterior lobe were 20, 21, 21, and 13 cases, respectively; and 38 cases of admission combined with shock. There was no statistical difference between the two groups in gender, age, tumor diameter, and other general data. The hospital ethics committee has reviewed and approved this study. The patients and their families were aware of this study and signed the informed consent.

### 2.2. Methods

1. The patients in the TAE group were placed in a supine position. After sterilizing and laying a towel, lidocaine was injected into the femoral artery puncture point for local anesthesia. The femoral artery was punctured first, and a catheter was placed in the celiac trunk. The tumor in the right lobe of the liver is heavily stained with a contrast agent. The catheter was introduced to the proximal end of the common hepatic artery, a microcatheter and a microguide wire were inserted, and the microcatheter was introduced into the tumor supplying artery of the right hepatic artery, which was confirmed by angiography. A mixture of chemotherapeutic drugs such as carboplatin and an embolic agent was slowly injected, and the angiography showed that the blood supplying artery was well embolized, and no tumor was supplied by the artery. The microcatheter was introduced into another feeding artery, and super-liquefied lipiodol and an appropriate amount of 1-2 mm gelatin sponge particles were used for embolization in the same way until all the feeding arteries were embolized; final angiography in the right hepatic artery: no tumor staining. At the end of the operation, the catheter was removed and the groin was bandaged.
2. Combination group underwent elective partial hepatectomy after TAE, choosing different positions according to the location of the tumor. After continuous epidural anesthesia and combined anesthesia with endotracheal intubation, an oblique incision was made 1-2 transverse fingers below the right costal margin, and the abdominal organs and tumors are explored after laparotomy. Depending on the location of the tumor, the hepatic ligament was selectively dissociated to fully expose the tumor. The first hepatic hilum needed to be blocked according to the actual situation during the operation. The liver capsule and superficial liver tissue, blood vessels were incised with electrocautery at a distance of more than 2 cm from the tumor edge. The liver tissue was separated with forceps, and the tumor was completely removed after cutting off each duct. The stump of the duct was carefully ligated, and the large duct was sutured. The liver section was closed and sutured. The surgical field was flushed with normal saline, and a latex tube was placed under the right diaphragm or in the surgical area for drainage.

### 2.3. Observation Indicators

1. The operation-related indicators of the two groups were observed and counted, as well as the number of patients with successful hemostasis and the number of patients with lesion resection. The success of hemostasis was judged according to whether the clinical symptoms of the patient were relieved and whether the biochemical indicators such as hemoglobin, blood pressure, and the basic vital signs were stable.
2. Comparing the hemostatic effects of all patients by using Mindray DC-N2S Doppler ultrasonography to detect hemodynamic indexes, mean arterial pressure (MAP), and heart rate (HR), the 7060 automatic biochemical analyzer was used to detect the hemoglobin level.
3. Liver function indexes used ethylenediaminetetraacetic acid anticoagulation tube to collect 5 mL of fasting venous blood before and after surgery, centrifuged at 3000 r/min for 10 min, and took the upper serum part after separation, using 7060 automatic biochemical analyzer to detect blood biochemical indicators, including serum alpha-fetoprotein (AFP), albumin (ALB), and total bilirubin (TBIL).
4. During hospitalization, the occurrence of complications (pulmonary embolism, secondary hemorrhage, bile leakage in liver section, and pulmonary infection) in the two groups were observed and recorded.
5. All Patients were followed up by telephone or outpatient visits every 3 months after surgery. The deadline for follow-up is February 2022. The follow-up time ranged from 1 to 12 months. The survival rate and recurrence rate were compared between the two groups. The survival rate was judged based on whether the patient had a liver cancer-related death. The presence of liver cancer recurrence and ruptured hemorrhage was judged based on whether the patient had abdominal symptoms, whether there were abnormal changes of tumor markers *α*-fetoprotein, routine blood tests, liver function, and other laboratory indicators, and whether there were changes in imaging examinations.

### 2.4. Statistical Methods

All counting and measurement data were processed by using SPSS 22.0 for statistical data analysis, Shapiro–Wilk was used for measurement data for normality test, and the data satisfying normal distribution was expressed in the form of ($\bar{x}\pm s$). Independent *t*-test and paired *t*-test were used to compare the differences between groups and within groups, respectively, and the data that did not meet the normal distribution were expressed in the form of *M* (P25, P75), and the Kruskal–Wallis H rank sum test was used; the count data were expressed by the number of cases or rates, and the *χ*^2^ test was used to compare differences between groups; Kaplan–Meier was used for analysis of postoperative 1-year survival rate, log-rank test was used as well. Statistical value *P* < 0.05 indicates that there is statistical significance.

## 3. Results

### 3.1. Comparison of Surgery-Related Indicators between the Two Groups

Compared with the TAE group, the combination group had a shorter hospital stay, higher hemostasis success rate, and higher lesion clearance rate (*P* < 0.05), and the above differences were statistically significant (*P* < 0.05), as shown in Table 1.

### 3.2. Comparison of Hemostatic Effects between the Two Groups

There was no significant difference in MAP, HR, and hemoglobin between the TAE group and the combination group before the operation (*P* > 0.05); after the operation, the HR levels of the two groups were significantly decreased, the MAP and hemoglobin levels were significantly increased, and the HR of the combination group was significantly increased. The levels were lower, and the levels of MAP and hemoglobin were higher, and the above differences were statistically significant (*P* < 0.05), as shown in Figure 1 and Table 2.

### 3.3. Comparison of Liver Function Indicators between the Two Groups

There was no significant difference in the liver function indicators (AFP, ALB, and TBIL) between the TAE group and the combination group before operation (*P* > 0.05); the serum AFP levels of the two groups after operation were significantly decreased, and the serum ALB and TBIL levels increased significantly. The serum AFP level in the combination group was lower, while the serum ALB and TBIL levels were higher, and the above differences were statistically significant (*P* < 0.05), as shown in Figure 2 and Table 3.

### 3.4. Comparison of Postoperative Complications between the Two Groups

There was no significant difference in the incidence of postoperative complications (including pulmonary embolism, secondary hemorrhage, bile leakage in the liver section, and pulmonary infection) between the TAE group and the combination group (*P* > 0.05), as shown in Table 4.

### 3.5. Comparison of 1-Year Survival Rate and Recurrence Rate between the Two Groups

A one-year follow-up showed that 20 patients in the combination group died due to liver cancer, and 35 patients in the TAE group died due to liver cancer. The 1-year overall survival rate in the combination group (73.33%) was significantly higher than that in the TAE group (53.33%), as shown in Figure 3. Compared with TAE group (40.00%), the combination group (17.33%) had a lower recurrence rate and a higher survival rate at 1 year after operation, and the above differences were statistically significant (*P* < 0.05), as shown in Table 5.

## 4. Discussion

The global incidence of primary liver cancer is increasing, ranking third in the mortality risk of malignant tumors, and it accounts for 80% of hepatocellular carcinoma, which seriously threatens human health and life [8]. The incidence of primary liver cancer rupture and hemorrhage is 10% to 20%. Clinically, it is one of the main causes of death in patients with primary liver cancer [9, 10]. TAE belongs to minimally invasive interventional therapy. It can be used not only for the treatment of liver hemorrhage but also for the treatment of primary liver cancer. Previous studies [11, 12] reported that TAE has a good short-term effect in the treatment of primary liver cancer, and it can be less interventional in the number of embolizations, but when the tumor diameter exceeds 10 cm, TAE is less effective. Liver resection is the preferred option and the key to improving patient survival. Relevant studies [13, 14] reported that partial hepatectomy can shorten the recovery time of patients and reduce the recurrence rate of patients after surgery. Therefore, this study selected patients with ruptured hemorrhage of primary liver cancer to undergo partial hepatectomy after TAE.

This study found that compared with the TAE group, the combination group had a shorter hospital stay, a higher rate of successful hemostasis and a higher rate of lesion clearance. For resectable primary liver cancer, partial hepatectomy is still a good treatment, not only for surgical hemostasis but also for radical resection of the tumor. The clinical efficacy is obviously superior to that of conservative treatment or simple intervention treatment [15]. Combined with the above reports, this study suggests that partial hepatectomy for primary liver cancer rupture and bleeding after TAE can improve the hemostatic effect and lesion clearance rate of TAE treatment and improve the short-term efficacy of patients. At the same time, this study found that the HR levels of the two groups of patients after surgery were significantly decreased, and the levels of MAP and hemoglobin were significantly increased, and the combination group had lower HR levels and higher MAP and hemoglobin levels, which further confirmed that partial hepatectomy for ruptured hemorrhage of primary liver cancer after TAE can improve the hemostatic effect.

Liver failure is one of the most serious complications after liver cancer resection, and its main clinical manifestations include obvious hypoalbuminemia and hyperbilirubinemia [16]. Hyperbilirubinemia is mainly due to the destruction and hemolysis of red blood cells caused by various reasons such as blood absorption in the interstitial space caused by surgery [17]. Hypoalbuminemia is mainly due to excessive intraoperative consumption and untimely nutritional supply, resulting in decreased albumin [16]. This study found that the serum AFP levels of the two groups of patients after surgery were significantly decreased, and the serum ALB and TBIL levels were significantly increased. It is suggested that partial hepatectomy for primary liver cancer rupture and hemorrhage after TAE can effectively protect the liver function of patients. The reason may be that TAE pretreatment can control the growth and rupture and hemorrhage of liver cancer, reduce the difficulty of partial hepatectomy, and thus reduce intraoperative liver damage. And partial hepatectomy did not increase the incidence of postoperative complications, suggesting that partial hepatectomy after TAE is safe for ruptured hemorrhage of primary liver cancer. This study found that the combination group had a lower 1-year recurrence rate and a higher survival rate. Previous studies [18] reported that the application of TAE in the treatment of hepatic hemangioma has the characteristics of less trauma and low risk but combined with liver resection can improve the treatment effect and also have a significant effect on improving the long-term survival rate of patients. Some studies [19, 20] found that for resectable ruptured hemorrhage of primary liver cancer, TAE combined with two-stage liver resection can significantly reduce perioperative complications, mortality, and improve patient survival. The results of this study combined with the above reports suggest that partial hepatectomy for ruptured hemorrhage of primary liver cancer after TAE can reduce the postoperative recurrence rate improve the prognosis and survival rate and has a good long-term effect.

In conclusion, partial hepatectomy after TAE in the treatment of ruptured hemorrhage of primary liver cancer can effectively improve the hemostatic effect, protect the liver function, improve the prognosis and survival rate, and reduce the postoperative recurrence rate. However, there were still some deficiencies in this study. For example, it was a single-center study with a small number of samples, and there may be some data biases. In the later stage, further multicenter and large-sample clinical trials are needed for in-depth research.

## Figures and Tables

**Figure 1:** Level distribution of postoperative hemostatic effect-related indicators in the two groups. (a) Level distribution of postoperative hemostatic effect-related indicators in TAE group; (b) level distribution of postoperative hemostatic effect-related indicators in combination group.

**Figure 2:** Level distribution of postoperative liver function-related indicators in the two groups. (a) Level distribution of postoperative liver function-related indicators in the TAE group; (b) levels of postoperative liver function-related indicators in the combination group.

**Figure 3:** Comparison of 1-year overall survival rate between TAE group and combination group.

**Table 1:** Comparison of surgery-related indicators between the two groups ($\bar{x}\pm s$, *n* (%)).

Group	Case	Hospital stay (*d*)	Hemostasis success rate (%)	Lesion clearance rate (%)
TAE	75	6 (5, 7)	62 (82.67)	55 (73.33)
Combination	75	6 (6, 7)	73 (97.33)	74 (98.67)
*Z*/*χ*^2^		−1.629	8.963	19.989
*P*		0.103	0.003	<0.001

**Table 2:** Comparison of hemostatic effects between the two groups ($\bar{x}\pm s$).

Group	Case	MAP (mmHg)		HR (Time/min)		Hemoglobin (g/dL)	
		Preoperative	Postoperative	Preoperative	Postoperative	Preoperative	Postoperative
TAE	75	71.94 ± 7.96	80.86 ± 9.88^*∗*^	129.02 ± 15.16	93.29 ± 10.67^*∗*^	7.13 ± 0.76	9.31 ± 1.14^*∗*^
Combination	75	72.46 ± 9.11	90.51 ± 11.33^*∗*^	129.03 ± 15.84	88.12 ± 10.75^*∗*^	7.33 ± 0.92	11.56 ± 1.34^*∗*^
*t*		0.372	5.583	0.004	2.956	1.451	11.076
*P*		0.710	<0.001	0.997	0.004	0.149	<0.001

Compared with the same group before operation, ^*∗*^*P* < 0.05.

**Table 3:** Comparison of liver function indicators between the two groups ($\bar{x}\pm s$).

Group	Case	AFP (*μ*g/L)		ALB (g/L)		TBIL (*μ*mol/L)	
		Preoperative	Postoperative	Preoperative	Postoperative	Preoperative	Postoperative
TAE	75	529.42 ± 82.15	264.11 ± 35.34^*∗*^	30.58 ± 5.52	48.63 ± 5.54^*∗*^	10.26 ± 1.49	17.33 ± 2.10^*∗*^
Combination	75	520.76 ± 86.87	135.92 ± 23.13^*∗*^	30.88 ± 4.58	53.28 ± 6.03^*∗*^	10.43 ± 1.89	19.51 ± 1.91^*∗*^
*t*		0.627	26.284	0.362	4.918	0.612	6.651
*P*		0.531	<0.001	0.718	<0.001	0.542	<0.001

Compared with the same group before operation, ^*∗*^*P* < 0.05.

**Table 4:** Comparison of postoperative complications between the two groups (*n* (%)).

Group	Case	Pulmonary embolism	Secondary bleeding	Liver section bile leakage	Lung infection	Complication rate
TAE	75	5 (6.67)	2 (2.67)	0 (0.00)	3 (4.00)	10 (13.33)
Combination	75	2 (2.67)	0 (0.00)	1 (1.33)	1 (1.33)	4 (5.33)
*χ* ^2^						2.836
*P*						0.092

**Table 5:** Comparison of in-hospital mortality, 1-year survival rate, and recurrence rate between the two groups (*n* (%)).

Group	Case	1-year survival rate after surgery	1-year recurrence rate after surgery
TAE	75	40 (53.33)	30 (40.00)
Combination	75	55 (73.33)	13 (17.33)
*χ* ^2^		6.459	9.422
*P*		0.011	0.002

## Data Availability

The data can be obtained from the author upon reasonable request.
